The article "A Semantic-Based Approach for Managing Healthcare Big Data: A Survey" was published in 2020. Journal: J Healthc Eng.

# A Semantic-Based Approach for Managing Healthcare Big Data: A Survey

**DOI:** 10.1155/2020/8865808

**Published:** 2020-11-23

**Authors:** Rafat Hammad, Malek Barhoush, Bilal H. Abed-alguni

**Affiliations:** Yarmouk University, Irbid, Jordan

## Abstract

Healthcare information systems can reduce the expenses of treatment, foresee episodes of pestilences, help stay away from preventable illnesses, and improve personal life satisfaction. As of late, considerable volumes of heterogeneous and differing medicinal services data are being produced from different sources covering clinic records of patients, lab results, and wearable devices, making it hard for conventional data processing to handle and manage this amount of data. Confronted with the difficulties and challenges facing the process of managing healthcare big data such as volume, velocity, and variety, healthcare information systems need to use new methods and techniques for managing and processing such data to extract useful information and knowledge. In the recent few years, a large number of organizations and companies have shown enthusiasm for using semantic web technologies with healthcare big data to convert data into knowledge and intelligence. In this paper, we review the state of the art on the semantic web for the healthcare industry. Based on our literature review, we will discuss how different techniques, standards, and points of view created by the semantic web community can participate in addressing the challenges related to healthcare big data.

## 1. Introduction

Big healthcare data refers to the process of collecting, integrating, managing, processing, and analyzing different kinds of medical data, which are excessively complex and inefficient to be processed and managed using existing database management systems and tools [1–3]. Big data outperforms conventional systems in the amount of data and processing capacity. There are many definitions available for big data; the most recognized is the definition that was given by Douglas Laney [4], who presented three features of big data: volume, velocity, and variety (known as the 3 Vs). Many researchers have introduced other Vs to this definition [5], but the 3 V definition model stays the most widely accepted definition.

Volume refers to the amount of data generated by different information systems. Velocity refers to the speed at which data are being produced, processed, stored, and analyzed [6]. Variety refers to the types of data being captured and processed, which can have different degrees of organization (e.g., structured, unstructured, and semistructured) and different formats (e.g., plain text, video, audio, and images).

### 1.1. Motivation for This Survey

The data generated from biomedical research and the process of digitization the healthcare sector have already generated and will continue to produce large amounts of data. This data is generated from different resources such as clinical records, hospitals, patient monitoring devices, medical images, and lab results. With the present continuously improving innovation of technologies, it has become simpler to gather, manage, and analyze these different types of medical data to infer meaningful insights. [7, 8]. For example, Santis et al. [9] used reverse engineering approaches with laser scans and surface texturing to evaluate shift and reduction of the tibiofemoral contact area after meniscectomy. Medical image management remains an energizing field of exploration and applications for healthcare and biomedical research. It includes all the techniques that provide the efficient storage, transmission, and retrieving of image data [10].

One of the significant difficulties in utilizing large data in healthcare is interoperability. Clinical information is spread across numerous sources administered by various districts, emergency clinics, and managerial divisions. The reconciliation of these information sources would require building up a new framework where all information suppliers integrate with each other. Data coming from different resources will have many challenges because of the irregularity in naming, structure, organization, and format. A significant prerequisite is to catch applicable information and make it broadly accessible and available in a clean and consistent configuration for easy integration with other information systems [7].

In the last few years, the semantic web was introduced by the World Wide Web Consortium (W3C) to enable a simpler method for searching, reusing, integrating, and sharing information [11]. Semantic techniques have demonstrated to be the most pertinent for comprehending and solving a lot of difficulties and challenges which face the healthcare big data community. This explains why many researchers and scientists are centered on finding semantic-based solutions for big healthcare data [12]. Semantic techniques have profited healthcare communities by improving their effectiveness and efficiency. The following are a few applications which list some of the motivations for using semantic techniques to allocate big data in the healthcare domain [13]:

- Allowing medical doctors to understand as plenty as they can about an affected person and as early in their existence as possible, to pick out up caution signs and symptoms of significant contamination as they rise.
- Allowing patients to wear medical smart devices to keep them away from hospitals. These devices produce considerable amounts of data, and analysts can use different big data tools to handle this large volume of data in real-time mode.
- Improving care personalization by analyzing all available healthcare data. This allows delivering the right treatment to the right patient at the right time.
- Allowing hospitals to enhance their security by monitoring any unusual changes in the network traffic to stop any cyber attacks.
- Monitoring patients with partial disabilities to analyze their activities and know their requirements for coexistence with the community.

### 1.2. Organization of the Paper

This paper is an endeavor to concentrate on the impact of consolidating healthcare big data with the semantic web to make it more intelligent. The remainder of the paper is organized as follows: Section 2 discusses the concepts of semantic modeling and ontology. The contribution of semantics to healthcare big data acquisition is discussed in Section 3.  Section 4 discusses the role of semantic techniques in integrating healthcare data. Semantic healthcare repositories are discussed in Section 5. Finally, our ﬁndings and concluding remarks are summarized in Section 6 and Section 7.

## 2. Background and Related Work

In this section, we study various ideas identified in managing healthcare big data and give broad insights concerning these ideas to assist readers with understanding the basic concepts introduced in this paper.

### 2.1. XML, RDF, SPARQL, and OWL Languages

Semantic modeling uses the following languages to represent and model the contained data: Extensible Markup Language (XML), Resource Description Framework (RDF), SPARQL, and Web Ontology Language (OWL) [14].

XML is a simple text-based markup language that defines a set of rules for representing and describing documents in a format that is both human-readable and machine-readable. It is one of the most widely used formats for sharing structured information between computers and between people [15].  Figure 1 shows a sample of XML document:

RDF is a language for representing information about resources on the Web. It was designed to provide a common way to describe information so it can be exchanged between different types of computers regardless of their operating systems or programming languages. RDF documents are written in XML and the language used by RDF is called RDF/XML. RDF identifies things using Uniform Resource Identifier (URI) and describes resources with properties and property values [16].  Figure 2 shows a sample of RDF which describes the resource “http://www.example.com/rdfsource.html.”

SPARQL is a semantic query language for retrieving and manipulating data stored in RDF format [17].  Figure 3 shows SPARQL query which returns the names and emails of every patient in the RDF dataset.

OWL is an ontology language designed to represent knowledge about things and the relations between these things. It includes a set of operators for forming concept descriptions that can be used to share knowledge between applications [18].

### 2.2. Big Data Platforms and Tools

To scale and accommodate a large amount of healthcare data, healthcare management systems must use distributed computing platforms. Many of the available distributed platforms are built on top of Apache Hadoop, which is considered the base. Hadoop is an open-source framework that was designed to support distributed storage and processing using simple programming models. It consists of two main components: HDFS and MapReduce. HDFS is a distributed file system that stores data on a cluster of machines. MapReduce is a computational model that spreads data and calculations over any number of servers in the cluster.

On the other hand, NoSQL, which simply means “not only SQL, was created especially as a distributed database framework where data can be stored in multiple processing nodes.

There are a large number of available NoSQL databases these days. Based on the used data model, these databases are usually divided into four categories and shown in Table 1.

The NoSQL database must have a set of features and characteristics to perform their work in a highly efficient way, especially when dealing with big data applications, and these characteristics are summarized as follows [28]:

- Horizontal scalable: NoSQL data need to spread their data among multiple servers; this data needs to be treated efficiently
- Data replication: NoSQL data need to be replicated to improve performance
- Suitable consistency model: NoSQL replicated data need to be consistent with suitable concurrency
- Simple graphical user interface: to attract NoSQL users, the GUI must be simple and easy to use, and all operations performed in SQL databases can be done in NoSQL databases easily and conveniently
- Powerful data store: the data stored must be close to the user, which increases performance
- Flexible attribute resizing: different records within the NoSQL database may have different attributes, and this feature helps to reduce the tables in a database to the minimum

The semantic model is a method for arranging and organizing data so that it can be interpreted by computers without human mediation. It is a conceptual model that incorporates semantics and relations to data [29, 30]. Ontology is used as a common representation of knowledge, and this gives the flexibility to share and reuse knowledge between distributed and heterogeneous systems and databases [31]. It is considered as one of the main building blocks of semantic modeling and it consists of the following components [32]:

- Classes represent sorts of things in the world. For example, the human “Leg” represents a class.
- Instances of classes are individuals fulfilling the classes' intension. For example, the sentence “My Leg” represents an instance.
- Relations between instances emerge from the interactions of individuals. For example, “My Leg Is Part of Me” is considered a relation.
- Axioms specify our knowledge of the domain. For example, we can conclude the following sentence: “Every Instance of Foot Is a Part of an Instance of Leg.”

### 2.3. Related Work

The area of managing healthcare big data has recently grabbed a lot of attention and has been taken into consideration.  Table 2 sums up the key related research papers including our survey. Among these related surveys, none of these papers address the managing of healthcare big data from semantic respective.

### 2.4. Ontologies for Healthcare Data

Many ontologies have been created in the context of the healthcare domain. The greater part of these ontologies has been made to a particular area in healthcare such as drug development, human disease, rehabilitation, and human hereditary [7]. The list of ontologies is consistently developing and increasing and many of them are available at BioPortal [39].  Table 3 includes some examples of available healthcare ontologies with their features.

## 3. Semantics for Healthcare Data Acquisition

Data acquisition is the method of gathering, extracting, and transforming data before storing it in the repository, which will be used later for analysis. The acquisition of big data is regularly controlled by the three Vs which include volume, velocity, and variety [12, 46].

Powerful analysis is based on storing the right information. The semantic technologies can be used in data acquisition to extract related and important data. This allows the process of discovering and excluding unnecessary information that contains errors or irregularities before storing it in its final repository [12, 47].

Most of the semantic techniques which are used in healthcare data acquisition are based on using ontologies to represent the healthcare data by following these three steps: (1) converting source data sets to RDF, (2) using ontologies to apply conversion business rules to the RDF data, and (3) loading the processed data into their final repositories.

Ding et al. [48] developed a semantic web portal that enables patients to access all their medical information such as prescription, lab results, doctors, and diseases. This portal allows users to effectively disclose, search, discover, and visualize semantic data easily and smartly. It also enables the process of transforming data from one format, such as relational databases, into an RDF format [7].

Data provenance is utilized for depicting data evolution, which records the entire data process, including all changes and transformations which have been applied to change data from one state to another [49]. Zhao et al. [50] introduced different methods for modeling, capturing, and querying provenance data by identifying mapping joins between data generated from different sources related to genomics. The authors show the utilization of named RDF graphs with various degrees of granularity to make provenance declarations about connected data [51].

The Ambient Assisted Living (AAL) system attempts to make better living conditions for older and disabled people. Forkan et al. [52] proposed a cloud-based solution called CoCaMAAL to handle the process of data gathering and processing in AAL systems. They used ontologies to enhance AAL services by providing a single virtual community that includes patients, devices, and computational servers. The proposed model implements a service-oriented architecture (SOA) for uniﬁed context generation. This is achieved by processing and integrating the collected sensor data by choosing the ideal fitting services using a context management system (CMS).

Jiang et al. [53] proposed a context-awareness wearable sensor system. The proposed solution can handle large amounts of data generated from the continuous monitoring of devices wearable by the elderly, sending alerts to the right people when necessary, and sending valuable information for analysis using big data solutions.

Tilahun et al. [54] presented a set of Web semantic, called Linked Open Data (LOD), to publish and connect public heterogeneous health data. All healthcare data were stored in RDF graphs where the triples are connected using the Silk, an open-source framework for integrating different data sources [7].

Michel Dumontier and Villanueva-Rosales [55] introduced their knowledge base structured using semantic technologies to capture pharmacogenomics and related information such as genes, medications, and therapeutic. They represented their semantic information using XML markup languages. Utilizing semantic techniques to capture and model neuroradiological knowledge in a head injury situation and using an ontology to retrieve clinical neurological from different data sets were studied by Garcia et al. [56].

Ullah et al. [57] introduced a Semantic Interoperability Model for Big-Information in IoT (SIMB-IoT) to convey semantic interoperability between data generated from different healthcare information systems. They used annotations for big data, stored the data in an RDF format, and used SPARQL to query the data from the RDF graphs. Yoon et al. [58] proposed a web-based automated extraction system, called DiTex to extract disease-related topics using natural language processing and semantic similarity ranking algorithms. Pacaci et al. [59] developed a semantic transformation approach to extract data from electronic health record systems by converting source datasets to RDF and then loading the processed data into their final repository.

## 4. Semantics for Healthcare Data Integration

Data can exist over numerous datasets, which requires data to be consolidated and merged using some common ﬁelds [12]. Data integration can be defined as the process of integrating data from various sources in a standard format, storing data in proper repositories, and providing a uniﬁed view of the data to be used for retrieval and analysis [60].

Using semantic techniques for data integration has become progressively pivotal and has gained a lot of consideration in both database and Web communities. The utilization of ontology as a data broker can make data integration easier in different ways, such as providing global concepts to represent data, automating the process of data integration, and providing the ability to query data semantically [61].

Ethier et al. [62] built up a core ontology to deal with semantic interoperability across heterogeneous biomedical datasets within TRANSFoRm project. This project was designed as an infrastructure for a learning healthcare system in European Primary Care. Keller et al. [63] proposed a semantic framework for consolidating heterogeneous air traffic data using a shared ontology, which is used to transform the original source data into a unified RDF representation. The integrated RDF store can then be queried using SPARQL to retrieve information semantically.

HBase is a NoSQL column-oriented distributed database that can store considerable amounts of data from terabytes to petabytes of data [64]. Kang et al. [65] used HBase repository, ontologies, and data mapping to develop a semantic big data model that integrates heterogeneous data from different resources. Yu et al. [66] presented a framework to integrate data that are continuously generated from different healthcare providers. They used Kafka, a real-time streaming framework, to collect the stream data and store it in NoSQL database. They developed a semantic lifting engine to generate the RDF triples and store it in the Virtuoso RDF repository. They used Apache Jena RDF semantic reasoning framework to analyze the data to find any health risks.

Using ontologies to automatically generate SQL statements during the data extraction process was studied by Mate et al. [67]. They introduced an ontology-based approach to represent concepts of medical data. Schoppenhauer et al. [68] developed a model called Ontology-Based Data Access (OBDA), which maps biomedicine classes and relationships to database entries by generating equivalent SQL statements to retrieve data from heterogeneous relational databases. The data can be retrieved using SPARQ queries, and the result data can then be available as materialized or virtualized RDF triples.

Livingston et al. [69] created a common ontology-based semantic model to integrate and query heterogeneous biomedical data sources. They devolved a knowledge base system called KaBOB (the Knowledge Base of Biomedicine), which integrates data from 18 different biomedical datasets that produce millions of RDF triples.

Manning et al. [70] developed a metadata ontology to extract knowledge from biological data using semantic techniques. The RDF triples were generated by mapping metadata from different datasets into this ontology. A user-friendly interface was implemented to provide the capability to answer complex queries and retrieve data from both RDF and RDBMS sources and then display the results.

Issa et al. [71] used the Apache spark framework with semantic modeling to integrate, store, process, and analyze sensor big data. An ontology is generated first based on Semantic Sensor Network (SSN) to model the use of the sensor data, and then large amounts of raw sensor data are transformed to semantic data using the resulting SSN-based ontology.

Liang et al. [72] developed an ontology that is used to integrate data from genes, symptoms, diseases, and phenotype. They extracted data from various sources into the ontology and performed semantic reasoning to help select the right medications that will be effective for some diseases such as bipolar and epilepsy.

Mapping very large and diverse datasets (stored in XML, KML, JSON, structured plain text ﬁles, or relational databases) into a common shared domain ontology was researched by Knoblock and Szekely [73]. Their methodology depends on extracting, modeling, and storing data in a system called Karma, which will perform their data integration, visualization, and analysis in a distributed environment over the whole dataset. Ruttenberg et al. [74] introduced Neurocommons prototype knowledge base for integrating and querying biomedical knowledge from numerous sources and disciplines. The prototype allows users to evaluate, showing the practicality, and scalability of the current semantic tools.

Chisham et al. [75] developed an RDF-based store framework, called CDAO, to store phylogenetic data. The developed framework provides a web service to allow programmers to access data in the store. The framework also contains a friendly user interface and visualization capabilities, which allows users to execute different kinds of domain-specific queries and view the results. CDAO also has the capability to import different formats such as PHYLIP, MEGA, NeXML, and NEXUS and store them in the store.

HL7 (Health Level 7) is a set of standards that were developed to enable the exchange of data between different healthcare information systems. On the other side, IEEE 1451 is a set of standards that are used in the context of sensor data to enable communication between different transducers. HL7 and IEEE 1451 have a different format, which makes the process of integration difficult between them. Kim et al. [76] implemented a simple software interface engine that can send and receive messages in IEEE 1451 and HL7 formats and provide interoperability between the two formats.

In the context of biological data science, computational analyses require integrating numerous datasets coming from different sources to enable data analysis and knowledge discovery. Garcia et al. [56] built a semantic web-based system called LinkHub, which extracts the graph of relationships between biological entities that are stored in different data sources including both RDF and relational datasets. The system provides various interfaces to interact with and query this graph data.

Integrating continuously changing biosciences data sources (because their schema changes over time) was studied by Marenco et al. [77] who developed a framework called Query Integrator System (QIS). The framework is based on an ontology server that maps data elements to concepts in an ontology. It includes different tools and utilities such as a graphical interface to design a distributed query.

Cheung et al. [78] implemented a web-based prototype that allows interoperability between different types of yeast genome data that have different formats. The prototype uses a native RDF database to store the integrated data generated from various heterogeneous data sources. It supports the mapping and conversion process of relational databases to RDF format. It also supports the retrieval of data from the RDF database stored using RDF-based queries.

## 5. Semantics for Healthcare Big Data Storage

The number of healthcare RDF data collections surpasses billions of triples and keeps continuously increasing beyond the performance capacity of traditional RDF management systems running on a single machine. In the last few years, big data techniques started to inspire researchers to develop new distributed methods to handle this large amount of emerging data. Big data management techniques can assist healthcare organizations to build knowledge-based systems to extract and infer meaningful insights from different data sets [79].

Most of the semantic techniques which are used in healthcare data storage are based on using the MapReduce paradigm, which was widely used to store and query healthcare data stored in Hadoop Distributed File System (HDFS). MapReduce is a distributed framework that is intended to scale up from one single machine to thousands of machines and to handle considerable amounts of data using simple programming models. Data is stored as RDF triple graph and SPARQL query language is used to retrieve and query the RDF store.

Rohloff and Schantz [80] used a MapReduce framework to implement a triple-store, called SHARD, which was built on top of Hadoop and deployed in Amazon EC2 cloud. SHARD was designed to be distributed and scalable and has the ability to store and query datasets with billions of triples. It stores the data as RDF triple graph and query data using SPARQL query language. Husain et al. [81] presented a framework which is able to handle a large amounts of RDF data stored in Hadoop Distributed File System (HDFS), a highly fault-tolerant system. A greedy approach algorithm was introduced to generate a query plan for answering SPARQL queries using Hadoop's MapReduce framework.

HBase is a column-oriented nonrelational distributed database, which is used to store RDF triples. Jena is a Java framework which was used to provide a programmatic interface for RDF, SPARQL, and ontologies. Khadilkar et al. [82] presented Jena-HBase which uses HBase and Jena framework to manage RDF datasets. The implemented framework supports end-users with APIs to store, query, and reason over large amounts of RDF data in a cloud-based environment.

Zeng et al. [83] introduced a distributed in-memory RDF management system, called Trinity.RDF, that physically models and stores RDF data in its native graph form. The proposed system is scalable and has the ability to handle large amounts of RDF data that could reach trillions of triples. Because the data is stored as a graph, the system supports large scope of complex graph analytics on RDF data and processes SPARQL queries efficiently.

Galarraga et al. [84] implemented Partout, a distributed framework to manage a large volume of RDF triples in a cluster of machines. The framework depends on dividing RDF triples into fragments, and based on the query log, assigning the fragments that are used with each other to the same node in the cluster. There is a central coordinator node that is accountable for distributing the RDF triples among the hosts and running SPARQL queries with the best execution plan.

Hose and Schenkel [85] presented a distributed SPARQL engine, called WARP, for a large scale of RDF datasets. The proposed engine is based on partitioning and replication of RDF triples across cluster nodes, enabling efficient query execution. Huang et al. [86] presented a scalable management system for RDF data which is based on the Hadoop MapReduce framework. The proposed architecture is based on using a graph partitioning algorithm to store triples that are close to each other on the same machine in the cluster. Partitioning RDF graphs in this way will reduce the amount of network communication greatly during query execution.

Lee and Liu [87] introduced a semantic hash partitioning framework, called SHAPE, which is based on applying a bassline hash partition on the RDF graph, and then replicating the vital triples only to improve the utilization of data access locality. The proposed method reduced the query execution time significantly by minimizing the internode communication during the query distributed processing.

Quilitz and Leser [88] implemented an engine, called DARQ, for querying data from multiple distributed RDF repositories using a simple interface, transparent to end-users. The implementation is based on using the Service Description Language (SDL), which is a set of standards provided by the semantic community. SDL enables the query engine to decompose SPARQL queries into subqueries, which will then be sent to the individual data sources and the results are integrated back to end-users.

Saleem et al. [89] implemented a comprehensive and open repository for storing biomedical information that will be used to categorize genetic mutations responsible for cancer. Their approach is based on transforming their data (more than 20 billion triples) into an RDF format, which will be distributed across multiple SPARQL endpoints. The data can be queried using a federated SPARQL query processing engine.

Harth et al. [90] presented an approach for executing queries over linked data, published as RDF triples. Their framework is based on building an index structure, called QTree, to summarize the content of RDF graph-structured source data. The generated index structure was used to answer conjunctive queries over linked data in an efficient way.

Vocabulary of Interlinked Datasets (VoID) is a RDF schema for representing metadata about RDF datasets. It is designed by the semantic web community to simplify the process of publishing, discovering, and querying on a graph of interlinked datasets [91]. Görlitz and Staab [92] proposed a framework, called SPLENDID, for querying distributed RDF data using statistical information obtained from the VoID. SPLENDID uses the generated statistics to build a good query execution plan to improve the SPARQL query execution performance.

Hammad and Banikhalaf [93] introduced a parallelization framework for storing and querying XML-based healthcare medical records in a distributed XML repository. They used MapReduce to execute certain types of queries called containment queries. Schwarte et al. [94] presented FedX, a framework that incorporates parallelization techniques to enable efficient querying of multiple distributed heterogeneous RDF datasets. During query execution, subqueries are generated and the execution plan is evaluated at the relevant node machines, reducing the remote intermediate requests, and, consequently, improving the query performance. The retrieved partial results are aggregated locally and returned to end-users.

Min et al. [95] used edge computing to propose a reinforcement learning ofﬂoading scheme which enables healthcare IoT devices to improve their computation performance while preserving user privacy. Their schema used a Dyna architecture to accelerate the learning speed process of the healthcare IoT devices.

## 6. Challenges and Future Research Directions

Research in the healthcare domain has grown fundamentally; many challenging problems remain to be solved regarding dealing with healthcare big data semantically. In this section, we feature some research challenges and opportunities to help different scientists and researchers know the issues that need to be solved and investigated in the healthcare domain. The challenges and opportunities are featured as follows:

- Data quality considerations: when it comes to big data, it is not just about volume; the successful semantic management systems must maintain the following five characteristics during the data integration step: accuracy, completeness, reliability, relevance, and timeliness. Unfortunately, most of the existing semantic healthcare systems were developed without maintaining all these quality characteristics during the data integration step. Moreover, these solutions were created and developed targeting an answer for a speciﬁc domain of medicinal services with a shortage of providing a complete and comprehensive semantic healthcare solution. Further research is required regarding assessing the quality of healthcare system. To build up credibility, healthcare data are progressively supposed to show that it has the required quality by automating the process of data quality assessment.
- Semantic metadata management: metadata management includes setting up strategies and cycles that guarantee data can be incorporated, referenced, shared, connected, investigated, and kept up to meet the interests of the corporation's stakeholders. Metadata is produced every time new data is generated, modified, or deleted. Metadata management for healthcare systems faces many challenges and issues that need to be resolved. Healthcare big data processing engine should have the capability to automate the process of discovering and selecting the most appropriate data sources based on predefined business rules. Different datasets may store the same data in multiple locations even if they have the same semantic meaning. The semantic processing engine should have the ability to select the right datasets based on different criteria and dimensions, such as query performance and data quality: accuracy, completeness, currency, and consistency.
- Managing uncertainty in healthcare big data: the massive amount of data collected from different healthcare sources such as wearable devices and online social media naturally contains a certain amount of uncertainty because of noise, irregularity, and missing information. On the other hand, the process of analyzing such collected uncertain data requires progressed explanatory methods for effectively anticipating future blueprints with high exactness and progressed dynamic procedures. Leaving the data with uncertainty will cause stakeholders to untrust any future results based on this data. Unfortunately, little work has been done in the area of uncertainty with semantic healthcare big data. New methods and procedures based on machine learning (ML) and natural language processing (NLP) must be introduced to design uncertainty data models. Integrating ML and NLP with semantic healthcare big data should have the ability to give more exact quicker, and adaptable outcomes for analyzers and decision-makers.
- Securing healthcare data using blockchain: precise and complete healthcare data are one important resource for patients. Any changes in data by cyber-attackers can cause dangerous health problems, such as giving incorrect medicines or therapies to patients. Therefore, the protection of privacy and securing medical data records have consistently been a worry for everybody during healthcare data administration. The rise of blockchain innovation carries novel ideas to secure healthcare data which are stored on the host servers. Further research is required since blockchain requires a lot of computational resources to create blocks, which is inapplicable for medical sensor devices.

## 7. Summary and Conclusion

The healthcare community is constantly generating massive, high-speed, heterogeneous, and disparate data that includes structured, semistructured, and unstructured. Many challenges are facing the process of managing healthcare data such as volume, velocity, and variety. Unfortunately, traditional information systems are not capable of exploiting such data powerfully and efficiently.

In the previous sections, we have reviewed existing solutions found in the literature related to semantic healthcare big data management from different perspectives including data acquisition, data integration, and data storage. We summarize our ﬁndings in Table 4.

Semantic web technologies have the opportunity to transform the way healthcare providers utilize technology to gain insights and knowledge from their data and make decisions. Both big data and semantic web technologies can complement each other to address the previous challenges and add intelligence to healthcare management systems. This paper reviews some of those challenges and discusses the role of semantic Web technologies in healthcare management systems. The review was conducted from four viewpoints. First, we reviewed some of the semantic ontologies which have been created and used by the healthcare community. Second, we reviewed the role of semantic technologies in extracting and transforming healthcare data before storing it in repositories. Third, we conducted a review of the different approaches for integrating heterogeneous healthcare data. Finally, we reviewed the different semantic methods and approaches for storing healthcare data in distributed environments.

In our survey, we found some issues and challenges that need to be answered regarding dealing with healthcare big data semantically. We reported these limitations and challenges, and we discussed some of the potential research directions. We intend to lead an exploratory study with some of the potential solutions for managing big healthcare data semantically [96].

## Figures and Tables

**Figure 1:** A sample of XML document.

**Figure 2:** A sample of RDF document.

**Figure 3:** A sample of SPARQL query.

**Table 1:** Categories of NoSQL data models.

Data model	Description	Platform/tools
Key-value	It represents and stores data as a collection of key-value pairs.	Aerospike [19]
		Redis [20]
		RocksDB [21]

Document-oriented	It represents and stores data as documents, such as XML and JSON.	MongoDB [22]
		CouchDB [22]
		PostgreSQL [23]

Graph	It represents and stores data as graph structures with nodes, edges, and properties.	Neo4j [24]
		AllegroGraph [24]
		ArangoDB [24]

Column	It is a type of the key-value data model, but it uses the notions of rows and columns. It is different from relational databases because the names and format of the columns in the same table can fluctuate from row to row.	HBase [25]
		Cassandra [26]
		Accumulo [27]

**Table 2:** Related research papers.

Paper	Year	Description
[12]	2018	This study presents an overview that compares different approaches for analyzing big data using semantic techniques. The comparison includes the description of every methodology in addition to its downsides. This paper did not cover the issues of capturing and managing data, it focuses only on the analytical part of big data.
[33]	2012	This study presented and compared different RDF storage solutions using a predefined set of characteristics. This study did not cover RDF storage from distributed respective which is needed by big data management.
[11]	2018	This study covered several approaches for integrating big data coming from different sources using semantic techniques. This study did not cover the issues capturing and storing the integrated data in its final target storage repository.
[34]	2018	This study is a review of the exploration subjects in the ﬁeld of the semantic web over its ﬁrst 20 years of presence. The study includes recognizing the primary current research trends, challenges, and future research directions in the area of semantic web and linked data.
[35]	2014	This study presented an overview of different frameworks and methodologies which are used to analyze big data in the healthcare domain. This paper did not cover the management part of healthcare big data.
[36]	2015	This study presented the benefits, opportunities, and challenges of using big data in the healthcare field. It also covers a set of applications and methodologies which are used by healthcare and the medical community.
[37]	2010	This research paper presented a framework that uses cloud computing to connect and share information across hospitals. The proposed solution used distributed resources (hardware and software) to process large amounts of medical images.
[38]	2016	This study presented an overview that summarized the challenges which face the big healthcare data in terms of volume, velocity, variety, and veracity. It proposed a systematic data-management pipeline approach for extracting, storing, analyzing healthcare data. This survey did not cover the data management from semantic respective.
Current study	2020	This study reviews the state of the art of semantic web technologies in healthcare management systems. It reviews the role of semantic technologies in extracting, integrating, and storing healthcare big data in distributed environments.

**Table 3:** List of some ontologies in healthcare domain.

Reference	Ontology	Description	Format	Classes	Properties
[40]	MedDRA	Used for data entry, information retrieval, analysis, and visualization. It covers drug development, health consequences, and malfunction of gadgets.	UMLS	73,429	18
[41]	DOID	Used to represent human illness.	OBO	12,694	15
[42]	PMR	Used for decision support in rehabilitation.	OWL	1,597	52
[43]	HP	Used to give an organized vocabulary for the phenotypic highlights experienced in human genetic and focus on monogenic diseases.	OBO	18,407	0
[44]	ATC	Used to classify drug's ingredients according to the organ on which they act and their chemical characteristics.	UMLS	6,358	3
[45]	ICF	Used to classify health domains: body, individual, and cultural points of view.	OWL	1,596	67

**Table 4:** References are organized by data acquisition, data integration, data storage, and semantic techniques.

Reference	Data acquisition	Data integration	Data storage	Semantic techniques	Solution
Ding et al. [48]	*X*	*X*	*—*	*X*	A semantic web portal that allows patients to access all their medical information
Zhao et al. [50]	*X*	*X*	*X*	*X*	An infrastructure prototype for modeling, capturing, and querying RDF provenance genomics data.
Forkan et al. [52]	*X*	—	*X*	*X*	A cloud-based solution to gather and process data in AAL systems.
Jiang et al. [53]	*X*	*X*	—	—	A context-awareness system to handle a large amount of generated data from wearable healthcare devices.
Tilahun et al. [54]	—	*X*	*X*	*X*	Linked open data (LOD) to publish and connect public heterogeneous health data.
Dumontier et al. [55]	*X*	—	*X*	*X*	Knowledge base structured to capture pharmacogenomics information and store them in XML format.
Garcia et al. [56]	*X*	*X*	—	*X*	Used ontologies to capture and integrate neuroradiological data.
Ullah et al. [57]	—	*X*	*X*	*X*	Integrated different healthcare data and used SPARQL to query the data from the RDF graphs.
Yoon et al. [37	*X*	—	—	*X*	Proposed DiTex to extract disease-related topics using natural language processing and semantic similarity ranking algorithms.
Pacaci et al. [59]	*X*	—	—	—	Used semantic techniques to extract data from electronic health record systems and store the data in RDF
Ethier et al. [62]	—	*X*	—	*X*	Developed TRANSFoRm project which uses ontologies to integrate biomedical datasets
Yu et al. [66]	*X*	—	*X*	*X*	Used kafka to collect healthcare stream data and store it in the NoSQL database.
Mate et al. [67]	*X*	—	—	*X*	Used ontologies to automatically generate SQL statements during the data extraction process for medical data.
Schoppenhauer et al. [68]	*X*	*X*	*X*	*X*	Developed a model that maps biomedicine classes and relationships to database entries. This model was used to extract data and store it as RDF triples.
Livingston et al. [69]	—	*X*	*X*	*X*	Devolved a knowledge base system called KaBOB to integrate data from many different biomedical datasets and store the results in RDF triples.
Liang et al. [72]	—	*X*	—	*X*	Developed an ontology that integrates data from genes, symptoms, diseases, and phenotype.
Chisham et al. [75]	—	—	*X*	*X*	Developed an RDF-based store framework, called CDAO, to store phylogenetic data.
Rohloff et al. [80]	—	—	*X*	*X*	Used a MapReduce framework to implement a distributed scalable RDF triple-store, called SHARD.
Galarraga et al. [84]	—	—	*X*	*X*	Implemented partout, a distributed framework to manage a large volume of RDF triples in a cluster of machines.
